RETRACTED

# Up-regulation of microRNA-497-5p inhibits colorectal cancer cell proliferation and invasion via targeting PTPN3

**DOI:** 10.1042/BSR20191123

**Published:** 2019-08-13

**Authors:** Sen Hong, Zhenkun Yan, Helei Wang, Lei Ding, Miaomiao Bi

**Affiliations:** 1 Department of Colorectal and Anal Surgery, The First Hospital of Jilin University, Changchun 130021, Jilin, China; 2 Department of Endoscopy Center, China-Japan Union Hospital of Jilin University, Changchun 130022, Jilin China; 3 Department of Gastrointestinal Surgery, The First Hospital of Jilin University, Changchun 130021, Jilin, China; 4 Department of Radiology, China-Japan Union Hospital of Jilin University, Changchun 130022, Jilin, China; 5 Department of Ophthalmology, China-Japan Union Hospital of Jilin University, Changchun 130022, Jilin, China

**Keywords:** Colorectal cancer (CRC), invasion, microRNA-497-5p (miR-497-5p), proliferation, protein tyrosine phosphatase non-receptor type 3 (PTPN3)

## Abstract

To investigate the role of microRNA-497-5p (miR-497-5p) in the tumorigenesis of colorectal cancer (CRC), the present study applied qRT-PCR to detect the expression level of miR-497-5p in both clinical samples and CRC cell lines. Furthermore, to specifically evaluate the carcinogenic role of miR-497-5p in CRC, the expression of miR-497-5p was monitored by transfecting with the mimics or inhibitors of miR-497-5p. Transwell assay as well as CCK-8 assay were used to determine the functions of miR-497-5p on cell invasion, migration and proliferation, respectively. miR-497-5p expression was remarkably down-regulated in clinical samples with cancer development as well as in CRC cell lines. Additionally, low miR-497-5p expression was remarkably correlated with higher TNM stage and lymph node metastasis of CRC patients. Up-regulation of miR-497-5p significantly inhibited proliferation, migration, and invasion of LOVO CRC cell line. Conversely, antagonizing miR-497-5p significantly promoted cell proliferation, migration and invasion. Mechanistic analysis revealed that miR-497-5p directly bound to its downstream target, protein tyrosine phosphatase non-receptor type 3 (PTPN3), whose aberrant expression partially reversed inhibition of cell proliferation and migration. Taken together, the present study elucidated the inhibitory role of miR-497-5p in CRC via targeting PTPN3, which potentiated miR-497-5p as a potential therapeutic target for combating CRC.

## Introduction

Colorectal cancer (CRC) emerges as one of the most common gastrointestinal malignancies and ranks second in cancer deaths worldwide [1]. Despite the advancement of diagnostic technologies and treatment management in the past decades, long-term survival rate in patients with CRC remains extremely low due to inadequate diagnosis and treatment in early stages of carcinoma [2–4]. At present, the molecular mechanism regarding hepatic metastases of colon and rectal carcinoma remains largely unknown. Therefore, it is of great significance to illuminate the molecular mechanism of CRC development and progression and further explore new molecular targets to diagnose and treat CRC in early stage.

RETRACTED

MicroRNAs (miRNAs) have approximately 21 nucleotides in length. And they are among one category of small noncoding RNAs and post-transcriptionally regulate genes expression via translational suppression as well as destabilization of target mRNAs [5,6]. Emerging evidence has implicated the regulatory roles miRNAs in cancer-related pathogenesis, acting as oncogenes or tumor suppressors [7,8]. Aberrant miRNA expression was found in various tumors, including prostate cancer, breast cancer, hepatocellular carcinoma, lung cancer as well as colon cancer, indicating the close relevance between miRNAs and malignant tumor [9]. Nevertheless, the role of miRNAs in the development of CRC is merely unknown.

Protein Tyrosine Phosphatase Non-Receptor Type 3 (PTPN3), also known as Protein Tyrosine Phosphatase H1 (PTPH1), belongs to the non-transmembrane PTP superfamily, which was initially identified in the cytosol and enriched at the plasma membrane in circulating T lymphocytes [14]. And it was tightly regulated in breast, glioma, colorectal and lung cancers [10–13]. A previous study found that PTPN3 was regulated by miR-199 in resistant ovarian cancer cells, suggesting that it is a potential therapeutic target for the ovarian cancer treatment [15].

Previous studies suggest that microRNA-497-5p (miR-497-5p) plays an oncogenic role in many tumor types [23]. Nevertheless, the comprehensive role and molecular mechanism of miR-497-5p in CRC have not been comprehensively studied yet. In the present study, the role and molecular mechanism of miR-497-5p in CRC development is explored, which may provide a potential solution to CRC diagnosis and treatment.

## Materials and methods

### Human CRC tissues samples

A total of 92 paired samples of human CRC and their matched adjacent normal individuals were collected from January 2011 to October 2013 in the China-Japan Union Hospital, Jilin University. None of the patients received radiotherapy or chemotherapy before surgery. All patients enrolled in this research signed the written informed consent. The study not only obtained approval of the Ethical Board of the Institute of China-Japan Union Hospital of Jilin University (approval number: CJUH19035), but also complied with the Declaration of Helsinki.

RETRACTED

### Cell culture

SW480, HT29, LOVO, SW620 human CRC cell lines were acquired from American Type Culture Collection (ATCC; U.S.A.) and they were maintained in RPMI 1640 (PAA, Gemany) supplemented with 10% fetal bovine serum (Hyclone, Logan, UT) and 100 U/ml penicillin (Life Technologies Corporation). Normal intestinal epithelial cells (NCM460) were cultured in Dulbecco’s modified Eagle’s medium (Gibco, Grand Island, NY, U.S.A.) supplemented with 10% fetal bovine serum (Gibco), streptomycin (100 lg/ml) as well as penicillin (100 U/ml) and incubated at 37°C in a humidified incubator with 5% CO_2_.

### Cell transfection

CRC cells were transfected with miR-497-5p mimics, inhibitor and scrambled mimics, which were synthesized by RiboBio (Guangzhou, China) via Lipofetamine 2000 Reagent transfection system (U.S.A.) according to the manufacturer’s instructions.

### qRT-PCR

Total RNA was extracted from CRC frozen tissue specimen as well as CRC cell line using TRIzol reagent (Invitrogen) by following the instructions. To assess expression of miR-497-5p, quantitative PCR was conducted on the Applied Biosystems (U.S.A.), In details, cDNA synthesis was first acquired using Superscript II reverse transcriptase (Invitrogen). qRT-PCR was then performed with a SYBR Premix Ex Taq™ II kit (TaKaRa). Primer sequences used for miRNA and mRNA expression analyses were as follows: miR-497-5p, F: 5′-AGCGAAGTTTTGAGCCGATCGGGC-3′, R: 5′-GCCGTGAGTCAGAGGTGGT-3′; PTPN3, F: 5′-GGCCTCGCATCCTCACGCT-3′, R: 5′-TGTGTATCGTTGCGGCGAATCCA-3′; GAPDH, F: 5′-CACGCGACCTTGGCTGTGT-3′, 5′-GTGAGGGCTTGGTCGGGATTGG-3′. The 2^−ΔΔ*C*^_t_ method was used to quantify the results and perform analysis. All reactions were run in triplicates.

### Cell proliferation

CCK-8 (Dojindo; Kumamoto, Japan) was used to incubate the cells as previously described [16]. The cell proliferative rates of CRC cells were determined at 0, 24, 48 and 72 h after transfection. Ten microliters of CCK-8 solution was added into each well and incubated for 2 h at 37°C. After that, numbers of viable cells were measured at the absorbance of 450 nm. The experiments were performed as triplicates.

### Scratch wound healing and Transwell assay

A wound healing assay was performed as previously described [17]. Transwell filter (BD Biosciences) was employed to perform Transwell invasion as previously described [18]. For the invasion assay, the transfected cells (2.5 × 10^5^) were plated in the top chamber with a Matrigel-coated membrane (BD Biosciences) in 500 μl serum-free DMEM accompanied by 750 μl of 10% FBS-DMEM in the bottom chamber. Non-invasive cells were taken out with cotton swabs, stained with Crystal Violet and counted under inverted microscope. After being stained with 0.1% Crystal Violet, the invasive cells located on lower surfaces of chambers were counted.

RETRACTED

### Dual luciferase reporter assay

PTPN3 3′UTRs containing forecast miR-497-5p target sites predicted via bioinformatics algorithms were amplified and cloned into pGL3-REPORT luciferase reporter vectors (U.S.A.). Constructed sequences containing wild-type PTPN3 3′UTR (PTPN3-WT) or mutations in putative target site of PTPN3 3′UTR (PTPN3-MUT) were obtained. The Lipofectamine 3000 (Invitrogen) was applied as transfection reagent for transfecting the recombined constructed pGL3-luciferase vector (U.S.A.) and miR-497-5p, or control mimic into LOVO cell. Plasmids of pGL3 with *Renilla* luciferase were used as internal control. The Luciferase reporter assay was performed with the Dual-Luciferase Reporter Assay System (Promega) based on manufacturer’s protocol. The whole transfection assays were performed in triplicate.

### Western blotting

Western blotting was performed by following the standard methods [19]. First, proteins were loaded on SDS/PAGE. After running, proteins in the gel were transferred on to PVDF membranes (Millipore, Bedford, MA, USA) by electrophoresis (Millipore, Billericay, Massachusetts). Then the membranes were blocked with 5% bovine serum albumin (BSA, Sigma–Aldrich, St. Louis, Missouri) for 1 h. Next, membranes were incubated with primary antibodies at 4°C overnight, which was followed by the secondary antibody incubation at room temperature for 1 h on the second day. The primary antibodies included anti-PTPN3 (1:1500, Abcam, Cambridge, MA, U.S.A.) and anti-GAPDH (1:1500, Santa Cruz Biotechnology). The secondary antibody was rabbit-anti-mouse IgG (1:2000, Santa Cruz Biotechnology, Santa Cruz, CA, U.S.A.). ECL Chemiluminescence Detection System (Thermo Fisher Science, Rochester, New York) was used to detect the chemical signal. The intensities of individual protein bands were quantified by Bio-Rad Quantity One software (Bio-Rad, Hercules, CA, U.S.A.). All procedures in the trial were repeated in triplicate.

### Hematoxylin and Eosin staining

Based on the triple-site gastric biopsy method, the histological diagnosis was performed as previously described [20]. After fixing in buffered formalin overnight, the organization was nested in paraffin. After that, 5.0 μm sections were selected for Hematoxylin and Eosin (H&E) staining (Sigma–Aldrich).

### Statistical analysis

The statistical analysis was carried out using SPSS 19.0 (SPSS Inc., Chicago, IL, U.S.A.). Data were presented as Mean ± SD. ANOVA or Student’s *t* test was used to compare the differences among multiple or two groups. The value of *P*<0.05 was considered as statistically significant difference.

RETRACTED

## Results

### Down-regulation of miR-497-5p in CRC tissues and cell lines

By comparison of the gene expression levels of miR-497-5p in CRC cell line SW480, HT29, LOVO, SW620 with that in normal intestinal epithelial cell line NCM460, miR-497-5p was significantly down-regulated in four CRC cell lines (*P*<0.001, Figure 1A). Furthermore, miR-497-5p expressions in 92 clinical primary CRC specimens and their adjacent para-carcinoma tissues were measured. H&E staining showed one representative pathological examination of CRC and para-carcinoma control tissues (Figure 1B). The result showed that miR-497-5p was down-regulated in 64 cases (77/92, 83.7%) (Figure 1C,D, *P*<0.001). Notably, miR-497-5p expression in CRC was negatively correlated with pTNM stage (*P*=0.004, Figure 1E). Nevertheless, no statistical relevance was found between miR-497-5p expression level and other clinical parameters (Table 1).

**Figure 1:** miR-497-5p expression in CRC tissues and cell lines (**A**) Pathological assay of representative CRC and adjacent matched-carcinoma tissues using H&E staining. (**B**) Relative gene expression level of miR-497-5p in CRC cell lines by comparison with NCM460 determined by qRT-PCR. (**C**) Relative expression of miR-497-5p in 92 primary CRC tissues compared with their matched-carcinoma tissues. (**D,E**) Association between miR-497-5p level with pTNM stage and metastases/non-metastases status. **P<0.01.

**Table 1:** Correlation of the expression of miR-497-5p in CRC with clinicopathologic parameters

Characteristics	miR-497-5p		*P*-value
	Low	High	
Age (years)			
<60	29	22	0.353
≥60	17	24	
Gender			
Male	38	16	0.678
Female	24	14	
Tumor size (cm)			
<5	23	20	0.081
≥5	39	10	
Lymph node metastasis			
No	19	11	0.469
Yes	43	19	
Differentiation			
Well and moderately	24	18	0.132
Poorly	38	12	
Depth of tumor			
T1 + T2	8	7	0.506
T3	10	12	
T4	28	27	
Tumor stage			
I + II	28	11	0.004
III	26	16	
IV	8	3	

### MiR-497-5p overexpression repressed CRC cell proliferation

Among these cell lines, the highest expression of miR-497-5p was detected in LOVO cell line, therefore it was chosen for further experiment. To explore whether miR-497-5p has inhibitory role in CRC, miR-497-5p mimics or inhibitor was transfected into LOVO cell line (Figure 2A). The growth curve showed that the proliferative rate of LOVO cell transfected with miR-497-5p mimic was significantly lower by comparison with those transfected with miR-NC. In contrast, LOVO cell transfected with miR-497-5p inhibitor increased proliferative rate (Figure 2B).

**Figure 2:** miR-497-5p overexpression suppressed CRC cell proliferation, migration and invasion (**A**) Expression levels of miR-497-5p after transfection with miR-497-5p mimics were detected by qRT-PCR. (**B**) Cells transfected with miR-497-5p mimics or inhibitors were examined by CCK8 assay. (**C**) Wound healing assays of LOVO cells were performed after cell transfection. (**D**) Transwell analysis of LOVO cells were performed after cell transfection. *P<0.05, **P<0.01 and ***P<0.001.

RETRACTED

### MiR-497-5p overexpression suppressed CRC cell migration and invasion

*In vitro* Transwell assays were performed to analyze the role of miR-497-5p on CRC cell migration and invasion. The data showed that the migrative ability of miR-497-5p mimics group cells was significantly lower than negative control group or untreated group. Inversely, miR-497-5p inhibitor remarkably increased migrative rate of LOVO cell (Figure 2C). Additionally, LOVO cell transfected with miR-497-5p mimics significantly increased the rate of cell migration by comparison with scramble group or untreated group. However, miR-497-5p inhibitor oligonucleotides remarkably enhanced the invasive rate of LOVO cell (Figure 2D). Taken together, miR-497-5p is a tumor suppressor in CRC cells.

### miR-497-5p directly targeted PTPN3 3′UTR in CRC cell

To search for the common set of putative targets of miR-497-5p, TargetScan (http://www.targetscan.org/vert_71/), miRDB (http://mirdb.org/) and miRanda (https://omictools.com/miranda-tool) were used. As predicted, the complementary sequence between miR-497-5p and PTPN3 3′UTR existed and was shown in Figure 3A. Then, the luciferase reporter assays were performed to explore the influence of miR-497-5p at PTPN3 mRNA level (Figure 3B). The results showed that ectopic miR-497-5p did not remarkably suppress the mutant PTPN3 3′UTR, but the luciferase activity of the WT reporter genes, which indicated that PTPN3 3′UTR was directly targeted by miR-497-5p. (Figure 3C,D). In clinical CRC samples (*n*=25), the statistically negative relation between PTPN3 and miR-497-5p level was also observed (two-sided Pearson correlation, r = −0.503, *P*=0.001, Figure 3E).

**Figure 3:** miR-497-5p targeted PTPN3 in gastric cancer cells (**A**) Sequences of miR-497-5p binding sites with WT/MUT PTPN3 3′UTRs. (**B**) Relative luciferase reporter activities of PTPN3-WT, PTPN3-MUT in LOVO cells. (**C**) PTPN3 mRNA expression in LOVO cells after treatment was detected by qRT-PCR analysis. (**D**) PTPN3 expression in LOVO cells after transfection was detected by Western blotting. (**E**) Bivariate correlation analysis of the association between PTPN3 expression and miR-497-5p levels. *P<0.05.

### Overexpression of PTPN3 reversed cell proliferation and invasion inhibition induced by miR-497-5p

Furthermore, the rescue assays were applied to confirm the role of PTPN3 in anti-tumor functions of miR-497-5p in CRC cells. It was demonstrated that miR-497-5p overexpression reduced PTPN3 protein level, which was reversed by pcDNA3.1-PTPN3 and miR-497-5p mimics co-transfection (Figure 4A). Meanwhile, overexpression of PTPN3 largely reversed the inhibitory effect of miR-497-5p on cell proliferation (Figure 4B). Furthermore, the inhibitory effects of wound healing and invasion induced by miR-497-5p overexpression were both markedly reversed by PTPN3 overexpression (Figure 4C,D). Thus, those results suggested that miR-497-5p exerted its tumor suppressive role via PTPN3. *In vivo*, PTPN3 protein level was negatively correlated with miR-497-5p level in CRC tissues by comparison with its adjoining non-tumor control organization (see Figure 5).

RETRACTED

**Figure 4:** Overexpression of PTPN3 reversed proliferation and invasion inhibition induced by miR-497-5p in CRC cells (**A**) Western blotting analysis of PTPN3 in LOVO cells co-transfected with either miR-497-5p mimic and pcDNA3.1-PTPN3. (**B**) OD 450 nm values of LOVO cells in different transfection groups. (**C,D**) Wound healing assay and Transwell analysis of LOVO cells in different transfection groups. *P<0.05 vs control group, #*P*<0.05 vs miR-497-5p group.

**Figure 5:** PTPN3 was up-regulated in CRC tissues PTPN3 expression was examined in eight miR-497-5p down-regulated CRC tissues and paired non-tumor tissues by Western blotting analysis.

## Discussion

Emerging evidence implied miRNAs’ critical roles in various cancer types, yet their expressions and functional roles in CRC remained poorly understood [21,22]. The present study revealed that the expression of miR-497-5p was remarkably down-regulated in CRC tissues as well as colon. Moreover, the expression of miR-497-5p expression was correlated with pTNM stage. miR-497-5p overexpression suppressed CRC cell proliferation, migration and invasion. Mechanistically, PTPN3 was identified as a direct indicator of miR-497-5p. In the study, miR-497-5p was found to act as a tumor suppressor in CRC tumorigenesis via inhibiting the proliferation, migration and invasion of cancer cells.

MiR-497-5p was reported to be overexpressed in angiosarcoma, melanoma and osteosarcoma previously [23–25]. In patients with non-small-cell lung cancer, miR-497-5p was related to lymph node metastasis and became the prognostic factor of metastasis as well as poor survival [26]. In addition, MiR-497-5p stimulated migration and infestation of melanoma A375 cells [25]. Our study has shown that miR-497-5p expression was significantly down-regulated in CRC specimen and clones. Moreover, reduced miR-497-5p expression was related to pTNM stage in clinical CRC patient tissues. Gain- and loss-of function studies were further applied to explore the function of miR-497-5p on biological behaviors of LOVO cells. It has shown that miR-497-5p dramatically supressed the proliferation, migration as well as invasion of LOVO cells, while the inhibitor of miR-497-5p significantly augmented the proliferation, migration and invasion abilities of LOVO cells. miR-497-5p restoration significantly repressed tumorigenic processes, indicating miR-497-5p restoration might be a potential therapeutic approach to treat CRC.

RETRACTED

By using bioinformatics tools, *PTPN3* was identified as the target gene regulated by miR-497-5p. Overexpression of miR-497-5p significantly reduced PTPN3 protein level and constrained PTPN3 3′UTR luciferase assay. Ectopic miR-497-5p failed to suppress mutant PTPN3 3′UTR but luciferase activity of WT reporter gene. PTPN3 was a well-acknowledged oncogene and was overexpressed in many types of tumors. It regulated genes participating in copious respects of tumorigenesis, like cell colony growth, resistance to apoptosis as well as angiogenesis [27,28]; cell transformation was induced by overexpression of PTPN3. Recent research has demonstrated that PTPN3 played a significant role in CRC growth and progression [12]. In our study, overexpression of PTPN3 significantly promoted LOVO cell proliferation and invasion. The present data revealed that miR-497-5p regulated gastric cancer via targeting PTPN3, rendering its underlining mechanisms for its post-transcriptional regulation.

## Conclusion

The present study elucidated the inhibitory role of miR-497-5p in CRC cell lines and clinical CRC samples. Moreover, *in vitro* study showed that overexpression of miR-497-5p suppressed CRC cell mass, infestation and transition via inhibiting PTPN3. The present study elucidates the role of miR-497-5-PTPN3 cascade in CRC carcinogenesis and potentiates miR-497-5p as a diagnostic biomarker and therapeutic target in CRC.

## Abbreviations

CCK-8: Cell counting kit-8
CRC: colorectal cancer
GAPDH: Glyceraldehyde 3-phosphate dehydrogenase
H&E: Hematoxylin and Eosin
miR-497-5p: microRNA-497-5p
pTNM: pathological tumor-nude-metastasis
PTPN3: protein tyrosine phosphatase non-receptor type 3
qRT-PCR: quantitative real time polymerase chain reaction
TNM: TNM classification of malignant tumors
